This article has been retracted.

# β_2_-adrenoreceptor Inverse Agonist Down-regulates Muscarine Cholinergic Subtype-3 Receptor and Its Downstream Signal Pathways in Airway Smooth Muscle Cells *in vitro*

**DOI:** 10.1038/srep39905

**Published:** 2017-01-04

**Authors:** Jian Luo, Yuan-hua Liu, Wei Luo, Zhu Luo, Chun-tao Liu

**Affiliations:** 1 Department of Respiratory Diseases, West China School of Medicine and West China Hospital, Sichuan University, Chengdu, 610041, China; 2 Department of Respiratory Diseases, The First Affiliated Hospital, Zhengzhou University, Zhengzhou, 450052, China; 3 Department of Respiratory Diseases, The First Affiliated Hospital, Chongqing Medical University, Chongqing, 400016, China

## Abstract

Mechanisms underlying β_2_-adrenoreceptor (β_2_AR) inverse agonist mediated bronchoprotectiveness remain unknown. We incubated ICI118,551, formoterol, budesonide, and formoterol plus budesonide, as well as ICI118,551 or pindolol plus formoterol, ICI118,551 plus forskolin, SQ22,536 or H89 plus formoterol in ASMCs to detect expressions of M_3_R, PLCβ_1_ and IP_3_. The level of M_3_R in the presence of 10^−5^ mmol/L ICI118,551 were significantly decreased at 12 h, 24 h and 48 h (P < 0.05), and at 24 h were significantly reduced in ICI118,551 with concentration of 10^−5 ^mmol/L, 10^−6 ^mmol/L, 10^−7 ^mmol/L, and 10^−8 ^mmol/L (P < 0.05). The level of IP_3_ in 10^−5 ^mmol/L ICI118,551 was significantly diminished at 24 h (P < 0.01), except for that at 1 h, neither was in the level of PLCβ_1_. A concentration of 10^−5 ^mmol/L ICI118,551 at 24 h showed a significant reduction of M_3_R level compared to formoterol (P < 0.01), budesonide (P < 0.01), and formoterol + budesonide (P < 0.05), but significant reduction of PLCβ_1_ and IP_3_ was only found between 10^−5 ^mmol/L ICI118,551 and formoterol at 24 h, but not in the comparison of budesonide or formoterol + budesonide. Pindolol and H89 could not inhibit the formoterol-induced expression of M_3_R (P > 0.05), but SQ22,536 significantly antagonized the formoterol-induced M_3_R expression (P < 0.05). In conclusions, β_2_AR inverse agonist, ICI118,551, exerts similar bronchoprotective effects to corticosteroids via decreasing the expression of M_3_R and inhibiting the production of IP_3_.

β-adrenoreceptor (βAR) agonists, especially β_2_-adrenoreceptor agonists, are the most common use bronchodilators in asthma treatment, and inhaled long-acting β_2_ agonists (LABA) are mainly used for long-term maintenance of symptoms relief as controller medications, of which salmeterol and formoterol account for the majority^1^. However, the adverse events of LABA gradually become significant clinical problems. Between 2008 and 2010, three alerts on LABA safety were made by American Food and Drug Administration (FDA), in which they pointed out the increased risk of exacerbation and mortality in asthmatic patients receiving long-term treatment of LABA^2^.

Similarly in previous debate in patients with congestive heart failure (CHF), in which βAR agonists were considered to be effective drugs due to their positive inotropic effects in increasing cardiac output but were revealed to increase mortality when used in a long-term fashion^3^,^4^, while βAR blockers were regarded as a contraindication based on their reduction of myocardial contraction but were validated to improve hemodynamics and attenuate mortality^5^,^6^, βAR blockers have always been listed as contraindications in asthma treatment, however, recent studies proposed potential benefits for patients with asthma and chronic obstructive pulmonary diseases (COPD) *in vitro*^7^,^8^,^9^. Furthermore, an open-label pilot study with 10 subjects showed that dose-escalating administration of βAR blocker, nadolol, exerted a significant and dose-dependent increase in provocation concentration of methacholine causing a 20% fall in forced expiratory volume in one second (PC_20_) (r = 0.86; p = 0.0016) although with a slight reduction in mean forced expiratory volume in one second (FEV_1_)^10^.

Moreover, different βAR blockers vary greatly in pharmacological properties. As demonstrated by a recent study^11^, a blocker could be roughly divided into antagonist and inverse agonist according to the presence of constitutive activity (or spontaneous activity) of a receptor and the degree of affinity and intrinsic activity of a ligand. Antagonists simply oppose the effects of agonists by preventing agonist binding and activation, while inverse agonists also reduce constitutive activity of the corresponding receptors besides the effects expressed by antagonists thus resulting in receptor activity inactivation beyond its baseline value. Studies have shown that β-blockers were inverse agonists and constitutive activity has been demonstrated in βAR^12^,^13^.

Nevertheless, the mechanisms underlying the asthma exacerbation induced by long-term use of LABA as well as the potential protective effects of βAR inverse agonists remain illusive. In our previous study, we found that continuous stimulation of airway smooth muscle cells (ASMCs) by formoterol up-regulated the expression of muscarine cholinergic subtype-3 receptor (M_3_R) via β_2_AR-cyclic adenosine monophosphate (cAMP)-phospholipase C (PLC)-inositol 1,4,5-trisphosphate (IP_3_) signal pathway thus resulting in reduction of bronchoprotective effects of formoterol^14^. Therefore, based on the assumption that overexpression of M_3_R and IP_3_ were in association with loss of bronchoprotective effects of LABA, we aimed to further investigate and validate the bronchoprotective effects of β_2_AR inverse agonist in ASMCs.

## Material and Methods

The study protocol was approved by the Biomedical Research Ethics Committee, West China Hospital, Sichuan University (Chengdu, China). All methods were performed in accordance with the relevant guidelines and regulations released by the Biomedical Research Center of West China Hospital.

### Reagents

ICI118,551 (a β_2_AR inverse agonist with high selectivity), pindolol (a β_2_AR non-inverse agonist), formoterol (a β_2_AR agonist), budesonide (a glucocorticoid), forskolin (a cAMP stimulator), SQ22,536 (a cAMP antagonist), and H89 (a PKA antagonist) were purchased from Tocris Bioscience (Bristol, UK). Acetylcholine (Ach, a cholinergic receptor agonist) was provided by Sigma-Aldrich (St. Louis, MO, USA).

Dulbecco’s modified Eagle’s medium (DMEM), fetal bovine serum (FBS) and 0.25% trypsin (containing ethylenediamine tetraacetic acid) were purchased from Gibco Life Technologies (Carlsbad, CA, USA). Rabbit polyclonal anti-α-smooth muscle actin antibody (cat. no. ab5694; 1:100 for immunocytochemistry and 1:2,000 for western blot analysis) and anti-M_3_R antibody (cat. no. ab41169; 1:100 for immunocytochemistry and 1:500 for western blot analysis) were purchased from Abcam (Cambridge, UK). A mouse polyclonal anti-rat anti-PLCβ_1_ antibody (cat. no. 610924; 1:1,000) was purchased from Becton Dickinson (Dublin, Ireland). Mouse anti-β‐actin and fluorescein isothiocyanate‐conjugated anti‐rabbit immunogobluin G (IgG) (cat. no. ZF‐0311; 1:100) antibodies were purchased from Zhongshan Golden Bridge Biological Technology Co. (Beijing, China). Horseradish peroxidase‐conjugated goat anti‐rabbit IgG (1:20,000) and goat anti-mouse IgG (1:20,000) secondary antibodies were obtained from Pierce (Rockford, IL, USA). The IP_3_ enzyme-linked immunosorbent assay (ELISA) kit was purchased from Cusabio Biotech Co., Ltd. (Wuhan, China).

### Primary rat ASMCs culture

Male Wistar rats (4 weeks old) were provided by the Animal Center of West China Hospital, Sichuan University (Chengdu, China). The rats were housed under specific pathogen free conditions at 25 °C and maintained on a 12-h light/dark cycle, with access to food and sterile water *ad libitum*.

Primary rat ASMCs cultures were prepared in accordance with the previously described methods^15^. After anesthetizing with 10% chloral hydrate, a total of 52 rats were sacrificed by cervical vertebra dislocation to obtain the tracheas, which were excised and minced in 10% FBS and DMEM, and the cells were allowed to adhere to the culture flasks for 3 h. Fresh culture medium (DMEM + FBS) was subsequently added and the cells were grown to confluence (density, 80 cells at ×200 high-power lens) in an incubator at 37 °C with 5% carbon dioxide (CO_2_). The cultured cells were then passaged following trypsinization with 0.05% trypsin, and ASMCs and their purity were detected by immunostained with anti-α‐smooth muscle actin antibodies in the third passage. Cells between fourth and sixth passage with > 80% confluence were used for subsequent experiments.

### Experimental procedures

ASMCs were incubated in the presence of various concentrations of ICI118,551 (10^−5^, 10^−6^, 10^−7^, and 10^−8 ^mmol/L) for 1, 6, 12, 24 and 48 h at 37 °C with 5% CO_2_, while the ASMCs cultured in DMEM + FBS only were defined as blank control. Expression levels of M_3_R were detected in different ICI118,551 concentrations at the incubation time of 24 h and at different incubation time in a ICI118,551 concentration of 10^−15 ^mmol/L, respectively, and the expression levels of PLCβ_1_ and IP_3_ were tested at the incubation time of 1 h and 24 h in a ICI118,551 concentration of 10^−5 ^mmol/L, after stimulation of 10^−4 ^mmol/L Ach for 15 min.

In addition, ASMCs were incubated with 10^−5 ^mmol/L formoterol, 10^−4 ^mmol/L budesonide, and 10^−5 ^mmol/L formoterol + 10^−4 ^mmol/L budesonide for 24 h, respectively, and were stimulated by 10^−4 ^mmol/L Ach for 15 min followed by detection of M_3_R, PLCβ_1_ and IP_3_ concentrations. Similarly, ASMCs were further incubated with 10^−5 ^mM ICI118,551 + 10^−5 ^mM formoterol, 10^−5 ^mM pindolol + 10^−5 ^mM formoterol, 10^−5 ^mM ICI118,551 + 10^−5 ^mM forskolin, 10^−4 ^mM SQ22,536 + 10^−5 ^mM formoterol, 10^−5 ^mM H89 + 10^−5 ^mM formoterol, and 10^−5 ^mmol/L formoterol for 24 h to detect the M_3_R levels after 15 min of Ach stimulation.

### Immunocytochemistry

The cultured cells (density, 80 cells at ×200 high-power lens) were fixed with 4% paraformaldehyde, blocked with goat serum (10%; Merck Millipore, Boston, MA, USA) and probed with primary antibodies specific to α-smooth muscle actin (1:100) (a smooth muscle cell specific marker) or M_3_R (1:100) overnight at 4 °C, followed by incubation with secondary antibody (1:100) at 37 °C for 1 h. The nuclei were stained with 4′,6-diamidino-2-phenylindole (Invitrogen, Carlsbad, CA, USA) for 5 min at room temperature. Images were captured using a confocal laser-scanning microscope (IX71-F22FL/PH, Olympus, Tokyo, Japan).

### Western blot analysis

The protein expression levels of M_3_R and PLCβ_1_ were measured by western blot analysis. The total cellular protein was extracted using radioimmunoprecipitation assay lysis buffer (1% Triton-X, 0.5% sodium deoxychlate, and 0.1% sodium dodecyl sulfate (SDS); Sangon Biotech, Shanghai, China), quantified using a bicinchoninic acid assay (Boster, Wuhan, China) and a Model 680 spectrophotometer (Bio-Rad Laboratories, Inc., Hercules, CA, USA), and adjusted to a concentration of 0.8 μg/μl. Equal quantities of protein were subjected to 5% sodium dodecyl sulphate polyacrylamide gel electrophoresis (12.6% separation gel for M_3_R, and β‐actin; 10% separation gel for PLCβ_1_; Sigma-Aldrich) and subsequently transferred onto polyvinylidene fluoride membranes (Merck Millipore). The membranes were blocked for 1 h with Tris-buffered saline containing 0.05% Tween-20 (TBST; Boster) and 5% goat serum (Boster) for M_3_R blots, or with 5% (w/v) non-fat milk for the PLCβ_1_ and β-actin blots. The membranes were subsequently incubated with primary antibodies against anti-M_3_R (1:500), anti-PLCβ_1_ (1:1,000) or anti-β-actin (1:2,000) at 4 °C overnight. Following incubation, the membranes were washed three times with TBST for 10 min and incubated with anti-rabbit (1:20,000) or anti-mouse (1:20,000) secondary antibodies for 1 h at room temperature. The membranes were subsequently washed and the blots were visualized using a Bio-Rad Gel DocTM XR + Imaging system and the band densities were quantified using Quantity One software (Bio-Rad Laboratories, Inc.).

### ELISA

The levels of IP3 were determined using an IP_3_ ELISA kit according to the manufacturer’s instructions. Briefly, the ASMC culture medium was removed and the cells were incubated with 0.1 mmol/l HClO_4_ for 20 min. The cells were centrifuged at 170 × g for 15 min at room temperature, and the supernatant was collected for analysis. An anti-IP_3_ detection antibody was added and incubated at 37 °C for 60 min, followed by the addition of substrate solution for 15 min at 37 °C. The reaction was terminated following the addition of stop solution and the plates were read at an absorbance of 450 nm to test the optical density (OD) value and calculate the IP_3_ concentration using a Model 680 spectrophotometer (Bio-Rad Laboratories, Inc.). The effect of ICI118,551 on the expression of IP_3_ was determined by the following formula: Inhibition of Ach-induced IP_3_ accumulation (%) = (IP_3_ levels in the control group − IP_3_ levels in the treatment group)/IP_3_ levels in the control group × 100%.

### Statistical analysis

Data are reported as the mean ± standard error of mean (SEM) and the differences between groups were analyzed using analysis of variance (ANOVA) and least significant difference (LSD). All statistical analyses were performed using SPSS 17.0 (SPSS, Inc., Chicago, IL, USA), and P < 0.05 was considered to indicate a statistically significant difference.

## Results

### Identification of rat ASMCs

The confluent rat ASMCs were arranged homogeneously in a multi-layered, polar fashion with the presence of “hill-and-valley” pattern (Fig. 1A). Immunofluorescence analysis showed the diffuse distribution of anti-smooth muscle actin within the cytoplasm in a fibroid profile, and the purification of ASMCs between the fourth and sixth passage was calculated to be >95% (Fig. 1B).

### Effects of different ICI118,551 concentration and incubation time on expression of M_3_R

Compared to the control ASMCs (0.5536 ± 0.0712), the level of M_3_R in the presence of 10^−5 ^mmol/L ICI118,551 were significantly decreased at 12 h (0.4073 ± 0.0605), 24 h (0.3394 ± 0.0674) and 48 h (0.3195 ± 0.0623) with a P value of < 0.05, but without significant differences at 1 h (0.5681 ± 0.0902) and 6 h (0.4975 ± 0.0768) with a P > 0.05 (Fig. 2).

As for the expression level of M_3_R in different ICI118,551 concentrations at 24 h, each ICI118,551 concentration presented a significantly lower M_3_R level (10^−8 ^mmol/L: 0.4682 ± 0.0647; 10^−7 ^mmol/L: 0.3826 ± 0.0764; 10^−6 ^mmol/L: 0.3511 ± 0.0517; 10^−5 ^mmol/L: 0.3468 ± 0.0563) than that in the control group (0.6311 ± 0.0658) with a P < 0.05 and a trend of dose-dependent manner (Fig. 3).

### Effects of ICI118,551 on expression of PLCβ_1_ and IP_3_

The level of PLCβ_1_ were slightly decreased in 10^−5 ^mmol/L ICI118,551 at 1 h (0.4937 ± 0.0767) and 24 h (0.5137 ± 0.0903) than that in control group (0.5522 ± 0.0694) but without significant differences (Fig. 4). The level of IP_3_ in 10^−5 ^mmol/L ICI118,551 at 1 h (6594 ± 902 pmol/L) was slightly higher than that in control group (6136 ± 1017 pmol/L), but significant difference was only found in the level of IP3 at 24 h (3085 ± 591 pmol/L, P < 0.01) (Fig. 5).

### Comparison of the effects of ICI118,551, formoterol, budesonide, and formoterol + budesonide on expression of M_3_R, PLCβ_1_ and IP_3_

A concentration of 10^−5 ^mmol/L ICI118,551 at 24 h showed a significant reduction of M_3_R level (0.3382 ± 0.0547) compared to formoterol (0.7299 ± 0.0716, P < 0.01), budesonide (0.4817 ± 0.0625, P < 0.01), and formoterol + budesonide (0.5741 ± 0.0608, P < 0.05) (Fig. 6A and B). However, significant reduction of PLCβ_1_ was only found between 10^−5 ^mmol/L ICI118,551 and formoterol at 24 h (0.5472 ± 0.0525 vs. 0.7335 ± 0.0594, P < 0.01), but not in the comparison of budesonide (0.5048 ± 0.0537) or formoterol + budesonide (0.5661 ± 0.0619) (Fig. 6C and D). A similar pattern was seen in level of IP3 with a significantly decreased IP3 level in 10^−5 ^mmol/L ICI118,551 at 24 h compared to that in formoterol (2694 ± 791 pmol/L vs. 4785 ± 853 pmol/L, P < 0.01) but an analogous level in budesonide (2536 ± 627 pmol/L) and formoterol + budesonide (3158 ± 534 pmol/L) (Fig. 6E).

### Comparison of the effects of ICI118,551/pindolol + formoterol, ICI118,551 + forskolin, SQ22,536/H89 + formoterol on M_3_R expression

Figure 7 depicted that a concentration of 10^−5 ^mmol/L ICI118,551 + formoterol at 24 h significantly reduced the M_3_R level compared to formoterol (0.4055 ± 0.0546 vs. 0.7442 ± 0.0756, P < 0.05), but pindolol + formoterol did not show any significant effect (0.6866 ± 0.0973 vs. 0.7442 ± 0.0756, P > 0.05). Pre-treatment with SQ22,536 significantly antagonized the formoterol-induced M_3_R expression (0.4903 ± 0.0708 vs. 0.7442 ± 0.0756, P < 0.05), however, we did not find a similar effect of H89 (0.5135 ± 0.0528 vs. 0.7442 ± 0.0756, P > 0.05). In addition, we noted that a concentration of 10^−5 ^mmol/L ICI118,551 could also inhibit the forskolin-induced expression of M_3_R (0.4273 ± 0.0502 vs. 0.7442 ± 0.0756, P < 0.05).

## Discussion

Since 1990 s, inhaled corticosteroids (ICS) with combination of LABA have been recommended as the first-line medication for asthma due to their efficacious bronchodilation and safety profile compared to short-acting β_2_ agonists (SABA). However, Nelson and his colleagues conducted a randomized, double-blind, placebo-controlled, observational study (SMART) in 26,355 subjects with asthma, and they revealed significant increase in respiratory-related deaths (24 vs. 11; RR 2.16; 95%CI 1.06 to 4.41) and asthma-related deaths (13 vs. 3; RR 4.37; 95%CI 1.25 to 15.34) in subjects receiving salmeterol compared to subjects receiving placebo^16^, which was further demonstrated in a meta-analysis with 19 trials containing 33,826 participants^17^. The increased exacerbation and mortality risk of LABA are recently suspected to be enhancement in bronchial hyperreactivity, airway inflammation and remodeling, and attenuation in bronchoprotective effects^9^,^18^.

Bronchoprotective effects are defined as anti-bronchoconstriction induced by various stimuli including allergen, exercise, cold air, histamine and Ach^19^. Chronic, regular use of β_2_AR agonists may induce tolerance to drug’s effects, in which bronchoprotection was found to be diminished or even lost rather than bronchodilation^20^,^21^,^22^,^23^,^24^,^25^. Furthermore, over-activation of β_2_AR can aggravate airway inflammation and airway responsiveness. Nguyen found reductions in lung mucous metaplasia, airway hyperresponsiveness (AHR), and inflammatory cells in β_2_AR-null mice^26^, while McGraw reported that β_2_AR overexpressing mice had enhanced constrictive responses to various stimuli^9^. In our previous study, we found that formoterol up-regulated M_3_R level by activating the β_2_AR-cAMP signaling pathway in a time- and dose-dependent manner and resulted in increased expression levels of PLCβ_1_ and IP_3_, which provided additional explanation for the loss of bronchoprotective effects induced by chronic use of LABA^14^.

It has been revealed that β agonists induced bronchodilation is the binding to the relaxed Gas-coupled receptors (mainly the β_2_AR), which results in decreased intracellular Ca^2 + ^through cAMP-dependent PKA induced phosphorylation of multiple proteins; while methacholine induced bronchoconstriction is targeting contractile Gaq-coupled receptors (including M_3_R), which triggers the release of Ca^2 + ^from sarcoplasmic reticulum via the activation of PLC and production of IP_3_^27^. Meanwhile, studies reported that a common physiologic consequence of chronic β_2_ agonist use is an increase in bronchoconstrictive responses to methacholine, which elucidated potential cross talk between the pathways of β_2_ agonists and methacholine. In our present study, we also found that cAMP inhibitor (SQ22,536) but not PKA inhibitor (H89) could significantly inhibit formoterol-induced up-regulation of M_3_R. However, the precise mechanisms have not been fully understood, but a reasonable consensus is that an adaptive program is in play so as to maintain bronchomotor tone or reactivity within a specific range^9^. Under this hypothesis, chronic or short-term use of β_2_ agonists may both break the balance and lead to hyperresponsiveness and bronchodilation. In addition, recent studies focused on the up-regulation of phosphodiesterase 4 (PDE4) by β_2_ agonists due to its degradation activity of cAMP, and they found that PDE4 mRNA was dose dependently up-regulated by fomoterol, which may serve as an alternative mechanism of β_2_ agonists induced loss of bronchodilation effects^28^.

Similar to the “paradoxical pharmacology” in CHF, βAR blockers have always been regarded as contraindication for asthma due to their pharmaceutical airway responsiveness exacerbation and bronchospasm. As a result, β_1_AR blockers with high selectivity are often prescribed for asthmatic patients with cardiovascular diseases such as metoprolol^29^. In fact, the selectivity of metoprolol is not as high as expected and the affinity to β_1_AR is reported to be only 2.3 times than that to β_2_AR^30^. On contrary, long-term use of βAR blockers have been found to be associated with small improvement in lung function and lower prevalence of respiratory adverse events in CHF with comorbidity of COPD or asthma^10^,^31^,^32^. Moreover, in rats asthma model, βAR blockers were demonstrated to alleviate airway inflammation and remodeling, and decrease bronchial hyperreactivity^33^,^34^. Therefore, βAR blockers have potential positive effects but are not the absolute contraindication in treatment of asthma.

Based on the constitutive activity (or spontaneous activity) of receptors, including G protein-coupled receptors (GPCRs), a ligand can be classified into 5 subgroups: full agonist, partial agonist, antagonist, partial inverse agonist, and full inverse agonist^11^,^35^,^36^. Inverse agonists have negative intrinsic activity and can reduce the spontaneous receptor activity due to the preferential binding and stabilizing receptors in the inactive state^37^. Nadolol and ICI118,551 are βAR inverse agonists and act as “gene knock out ” in pharmacology by silencing βAR via further blocking constitutive or spontaneous activity of βAR, while alprenolol, as a antagonist, do not have such an effect^38^. Therefore, not all βAR blockers can exert bronchoprotective effects as validated by the findings that attenuation in airway inflammation and hyperresponsiveness was only detected in asthmatic rats receiving nadolol and ICI118,551 rather than alprenolol, which was further demonstrated by our study with the comparison of ICI118,551 and a non-inverse agonist, pindolol^8^,^39^. Pindolol is a potent β2AR antagonist but lacks the effect of β2AR inverse agonist^13^,^40^. In our present study, we compared the M_3_R level among formoterol, pindolol + formoterol, and ICI118,551 + formoterol, and we found that M_3_R level was decreased in both pindolol + formoterol and ICI118,551 + formoterol group, but statistical significance was only detected in ICI118,551 + formoterol group. The reduction of M_3_R level in both pindolol + formoterol and ICI118,551 + formoterol group elucidated the involvement of β_2_AR in formoterol-induced M_3_R expression; while the statistically significant decrease of M_3_R level in ICI118,551 + formoterol group rather than pindolol + formoterol group further demonstrated the more important role of β_2_AR inverse agonist in blocking formoterol-induced M_3_R expression than simple β_2_AR antagonist.

Previoius hypothesis attributed the loss of bronchoprotection after chronic use of β_2_AR agonists to the reduction in β_2_AR synthesis and density over the cell surface by internalization, but it cannot completely explain the bronchoprotective effects induced by βAR inverse agonists in spite of an increase of lung βAR density after nadolol in rat asthma model^9^. Muscarine cholinergic receptors are also widely expressed in airway and are reported to mediate airway epithelial cells and hematopoietic cells in the regulation of airway inflammation in asthma^41^. In our present study, ICI118,551, as a βAR inverse agonist, significantly suppressed the expression of M_3_R at incubation time of 12 h and lasted for 48 h, and the degree of inhibition boosted as ICI118,551 concentration increased, which suggested that ICI118,551 could decrease the M_3_R expression in a time- and dose-dependent manner. However, the underlying mechanisms for such an influence of ICI118,551 on M_3_R expression still remains unknown, although recent findings suggested that interaction between arrestins and GPCRs desensitization/resensitization may play a role^41^.

From a pathophysiological view, airway smooth muscle tone and reactivity are regulated mainly by the GPCRs coupled to Gas and Gaq, of which GPCRs coupled to Gaq consist of M_3_R, thromboxane A_2_ (TXA_2_) receptor, 5-hydroxytryptamine (5-HT) subtype-2 receptor, cys-leukotriene recpetor, histamine receptor, platelet activating factor receptor and peptide receptor. Activation of GPCRs coupled to Gaq subsequently activates PLC and IP_3_, thus resulting in influx of Ca^2 + ^into cytoplasm and airway smooth muscle constriction. In our study, ICI118,551 significantly decreased level of IP_3_ at incubation time of 24 h compared to that at 1 h and that in control, which was similar to what reported in the experiment by Lin^42^. Our study result suggested that long incubation of ICI118,551 could reduce airway hyperresponsiveness and cell contractile signal to Ach. However, we did not find significant change of PLCβ_1_ after incubation with ICI118,551 either at 1 h or 24 h compared to control, which suggested that cell contractile signal decreased in a PLCβ_1_-independent way but necessitated further investigation.

As recommended by Global Initiative for Asthma (GINA) guideline, LABA should not be used as monotherapy in asthma, because ICS has been reported to not only suppress airway inflammation and hyperreactivity, however, it also prevent LABA induced down-regulation of β_2_AR and recover their sensitivity, thus may lead to increase of M_3_R, PLC-β_1_, and IP_3_ expression as demonstrated by McGraw^9^,^43^. On contrary, recent studies found that steroids could decrease the expression of muscarinic receptor and PDE4 mRNA in airway smooth muscle, which may result in bronchoprotection^28^,^43^,^44^,^45^. As a result, our present study did not show significant decrease of M_3_R, PLC-β_1_, and IP_3_ expression by budesonide compared with that by ICI118,551. On the other hand, chronic use of ICS also accompanied by potential adverse events, especially in asthmatic patients, including but not limited to blood glucose variation, osteoporosis, oropharyngeal fungal infections and pneumonia^46^, which forces clinicians to investigate novel medications to resist the adverse events caused by long-term use of β_2_AR agonists. Based on our previous findings that budesonide could significantly suppress the expression of formoterol induced M_3_R and PLCβ_1_ and IP3 exposed to Ach, we conducted this validation study of β_2_AR inverse agonist, ICI118,551, and the results showed pharmacological effects identical to budesonide but opposite to formoterol, which suggests the potential bronchoprotective effects of ICI118,551 and further demonstrates the findings reported previously^10^,^47^.

Recent pilot and randomized controlled trials showed inconsistent effects of different β_2_AR inverse agonists. Anderson randomly assigned 16 patients to receive propranolol 80 mg/d or placebo plus beclometasone 100 ug/d, and the results showed that histamine PC_20_ was unchanged and exhaled nitric oxide, blood eosinophils, serum eosinophilic cationic protein and asthma quality-of-life questionnaire symptoms were worsened by adding propranolol to beclometasone, which was further demonstrate by Short^48^,^49^,^50^. Therefore, inverse agonism as the key property for β-blockers is necessarily doubtful. Currently, ligand activation of the β_2_AR is recognized as the requirement for development of asthma^51^. β_2_AR has been shown to possess two independent signal pathways: the canonical Gs-AC-cAMP pathway and MAPKs like ERK1/2. The discrepancy in bronchoprotection effects of different β_2_AR inverse agonists is found to be attributed to the fact that propranolol is an inverse agonist at the Gs-cAMP signaling pathway and a partial agonist at ERK1/2 activation, while nadolol does not activate either of these signaling pathways^52^,^53^. However, our present study did not provide implications in such mechanisms, which might limit the recommendation of β_2_AR inverse agonists in treatment of asthma.

Additional limitations for our study included: 1) muscarine cholinergic subtype-2 receptor (M_2_R) was not investigated but it has been reported to constitute 80% of muscarinic receptors in ASMs, which might play a significant role in cross talk between β_2_AR. Future studies are warranted to target this receptor in exploring the mechanisms of β_2_AR inverse agonists; 2) in spite of the verified safety of βAR inverse agonist in the treatment of asthma, large amount of evidence-based and epidemiological data also showed that selective β-blockers are not completely risk-free. Morales reported that βAR inverse agonist may induce bronchospasm, impair lung function and worsen asthmatic symptoms regardless of selectivity^54^,^55^; 3) the potential influences of ASMCs passage number on M_3_R expression and the specificity of anti-M_3_R antibody we used should be further validated, which could bias the accuracy of our study; 4) the potential interaction of H89 on blocking β_2_AR besides PKA may result in ambiguous interpretations of our study outcomes, and future studies should use alternative PKA antagonist with high specificity and selectivity. Therefore, clinical application of βAR inverse agonists in patients with asthma should be cautious, and gradual increase from a low dose is recommended due to the consideration of safety profiles.

## Conclusions

β_2_AR inverse agonist, ICI118,551, exerts similar pharmacological effects to corticosteroids via decreasing the expression of M_3_R by GPCRs coupled to Gaq and inhibiting the production of IP_3_ induced by Ach, which provide a novel treatment strategy for patients with bronchial asthma, but future investigation of underlying mechanisms and validation of clinical implications *in vitro* and *in vivo* are warranted.

## Additional Information

**How to cite this article**: Luo, J. *et al*. β_2_-adrenoreceptor Inverse Agonist Down-regulates Muscarine Cholinergic Subtype-3 Receptor and Its Downstream Signal Pathways in Airway Smooth Muscle Cells *in vitro. Sci. Rep.* **7**, 39905; doi: 10.1038/srep39905 (2017).

**Publisher's note:** Springer Nature remains neutral with regard to jurisdictional claims in published maps and institutional affiliations.

## Figures and Tables

**Figure 1:** Primary culture of rat ASMCs. The primary culture of rat ASMCs were prepared. (**A**) Confluent cultured ASMCs were visualized under phase-contrast microscopy. (Magnification: ×200) (**B**) ASMCs were identified by immunocytochemistry staining with an anti-α-SMA antibody. Nuclear were double stained with DAPI. (Magnification: ×200). ASMCs, airway smooth muscle cells; DAPI, 4′,6-diamidino-2-phenylindole; SMA, smooth muscle actin.

**Figure 2:** ICI118,551 down-regulated the protein expression of M_3_R. (**A**) Cropped gel of M_3_R protein levels in rat ASMCs determined by Western blotting. The protein extract was obtained from ASMCs treated with 10^−5 ^mM ICI118,551 at indicated time points. (**B**) The densitometry results of M_3_R protein levels were normalized to β-actin control. Data were presented as means ± SEM from three independent experiments. DMEM + FBS served as control. ^*^Significant difference as compared to the control group (P < 0.05). ASMCs, airway smooth muscle cells; DMEM, Dulbecco’s modified Eagle’s medium; FBS, fetal bovine serum; M_3_R, muscarine cholinergic subtype-3 receptor; SEM, standard error of mean.

**Figure 3:** ICI118,551 dose-dependently down-regulated the protein expression of M_3_R. (**A**) Cropped gel of M_3_R protein levels in rat ASMCs determined by Western blotting. The protein extract was isolated from ASMCs treated with increasing doses of ICI118,551 for 24 h. (**B**) The densitometry results of M_3_R protein levels were normalized to a β-actin control. Data were presented as means ± SEM from three independent experiments. DMEM + FBS served as control. ^*^Significant difference as compared to the control group (P < 0.05). ASMCs, airway smooth muscle cells; DMEM, Dulbecco’s modified Eagle’s medium; FBS, fetal bovine serum; M_3_R, muscarine cholinergic subtype-3 receptor; SEM, standard error of mean.

**Figure 4:** ICI118,551 had no effect on the expression of PLCβ_1_. (**A**) Cropped gel of PLCβ_1_ protein levels in rat ASMCs determined by Western blotting. Rat ASMCs were randomly divided into control group, ICI118,551 1 h and 24 h groups, and received different treatments as described previously. (**B**) The densitometry results of PLCβ_1_ protein normalized to a β-actin control. Data were presented as means ± SEM from three independent experiments. DMEM + FBS served as control. There were no significant differences among the three group (P > 0.05). ASMCs, airway smooth muscle cells; DMEM, Dulbecco’s modified Eagle’s medium; FBS, fetal bovine serum; PLCβ_1_, phospholipase Cβ_1_; SEM, standard error of mean.

**Figure 5:** ICI118,551 suppressed the release of IP_3_ by Ach stimulation. The levels of IP_3_ were assayed by ELISA. DMEM + FBS served as control. ^*^Significant difference as compared with control group (P < 0.01). Ach, acetylcholine; DMEM, Dulbecco’s modified Eagle’s medium; FBS, fetal bovine serum; IP3, 1,4,5-trisphosphate; ELISA, enzyme-linked immunosorbent assay.

**Figure 6:** Comparison of the effects of ICI118,551, formoterol, budesonide/formoterol on M_3_R, PLCβ_1_ and IP_3_ expression. Rat ASMCs were randomly divided into five groups. Cells were incubated with 10^−5 ^mM ICI118,551, 10^−5 ^mM formoterol, 10^−4 ^mM budesonide, 10^−4 ^mM budesonide + 10^−5 ^mM formoterol and control group for 24 h. The M_3_R, PLCβ_1_ and IP_3_ levels were determined after 15 min of Ach (10^−4 ^mM) stimulation. Cropped gel of M_3_R (**A**) and PLCβ_1_ (**C**) protein levels in rat ASMCs were determined by Western blotting. The densitometry results of M_3_R (**B**) or PLCβ_1_ (**D**) were normalized to β-actin control. The expressions of IP_3_ were evaluated by ELISA (**E**). Data were presented as means ± SEM from three independent experiments. DMEM + FBS served as control. ^*^Significant difference as compared with 24 h of ICI118,551 treatment alone (P < 0.05). Ach, acetylcholine; ASMCs, airway smooth muscle cells; B, budesonide; F, formoterol; DMEM, Dulbecco’s modified Eagle’s medium; FBS, fetal bovine serum; ICI, ICI118,551; IP3, 1,4,5-trisphosphate; M_3_R, muscarine cholinergic subtype-3 receptor; PLCβ_1_, phospholipase Cβ_1_; SEM, standard error of mean.

**Figure 7:** Comparison of the effects of ICI118,551/pindolol + formoterol, ICI118,551 + forskolin, SQ22,536/H89 + formoterol, and formoterol on M_3_R expression. Rat ASMCs were randomly divided into seven groups. Cells were incubated with 10^−5 ^mM ICI118,551 + 10^−5 ^mM formoterol, 10^−5 ^mM pindolol + 10^−5 ^mM formoterol, 10^−5 ^mM ICI118,551 + 10^−5 ^mM forskolin, 10^−4 ^mM SQ22,536 + 10^−5 ^mM formoterol, 10^−5 ^mM H89 + 10^−5 ^mM formoterol, 10^−5 ^mM formoterol, and control group for 24 h. The M_3_R levels were determined after 15 min of Ach (10^−4 ^mM) stimulation. (**A**) Cropped gel of M_3_R protein levels in rat ASMCs determined by Western blotting. (**B**) The densitometry results of M_3_R protein levels were normalized to β-actin control. Data were presented as means ± SEM from three independent experiments. DMEM + FBS + formoterol served as control. *Significant difference as compared with 24 h of formoterol treatment alone (P < 0.05). Ach, acetylcholine; ASMCs, airway smooth muscle cells; DMEM, Dulbecco’s modified Eagle’s medium; F, formoterol; FBS, fetal bovine serum; FK, forskolin; ICI, ICI118,551; M_3_R, muscarine cholinergic subtype-3 receptor; P, pindolol; SEM, standard error of mean; SQ, SQ22,536.
